The article "Effects of Bisphosphonates on Osseointegration of Dental Implants in Rabbit Model" was published in 2021. Journal: Biomed Res Int.

# Effects of Bisphosphonates on Osseointegration of Dental Implants in Rabbit Model

**DOI:** 10.1155/2021/6689564

**Published:** 2021-02-12

**Authors:** Ru Qing Yu, Jing Yi Wang, Nian Jing Rao, Lei Huo, Li Wu Zheng

**Affiliations:** Discipline of Oral & Maxillofacial Surgery, Faculty of Dentistry, The University of Hong Kong, Hong Kong SAR, China

## Abstract

This study is to investigate the effect of bisphosphonates on the osseointegration of dental implants in a rabbit model. Twenty female New Zealand White rabbits were equally assigned into control and experiment groups which received saline or zoledronic acid treatment 4 weeks prior to surgery. Titanium dental implant was placed on the calvarial bone. Zoledronic acid or saline treatment continued after surgery for 4 weeks (short-term subgroup) or 8 weeks (long-term subgroup) until sacrifice. Three different fluorochrome labeling solutions were administrated for assessing bone growth rates. Samples of the calvarial bone and mandible were subjected to microcomputed tomography (micro-CT), confocal microscope, and histology analysis. Zoledronic acid treatment significantly reduced bone growth rates in the calvarial bone, but had no significant influence in bone mineral density and trabecular microarchitecture. Significantly lower bone-to-implant contact ratios were found in zoledronic acid-treated animals compared to controls at week 4 but not at week 8. Oncologic dose zoledronic acid suppresses the bone growth rates of the calvarial bone; ZA may have an adverse effect on osseointegration of dental implant in short term, but this effect tends to diminish in long term.

## 1. Introduction

Bisphosphonates work mainly on osteoclasts to reduce bone turnover rates and increase bone mineral density [1], mainly through their inhibitory effect on formation, differentiation, and activity of osteoblasts [2–7]. Bisphosphonates have been used to treat metabolic bone diseases, such as osteoporosis, Paget's disease, multiple myeloma, and bone metastasis [8]. Despite their great clinical benefits, a serious adverse event known as medication-related osteonecrosis of the jaws (MRONJ) has been reported.

Osseointegration is the principal success criteria of a dental implant [9], the concept of which was first discovered by Brånemark in 1969, demonstrating that it is a direct attachment between bone and the dental implant surface, with the competence of bearing the functional load [10]. Theoretically, the osseointegration of dental implants may benefit from bisphosphonates by reducing osteoclastic bone resorption and the subsequently diminishing bone remodeling; however, there is relatively limited data regarding the possible effects of bisphosphonates on relevant aspects of implant therapy, such as implant osseointegration, failure rate, and MRONJ development [11]. So far, there is no consensus concerning the placement of dental implants in patients receiving bisphosphonates. Most studies showed that low-dose oral BP for osteoporosis management does not compromise implant therapy, while there is almost no relevant information available on the possible effect on implant therapy of high-dose BPs [11].

The present study is aimed at evaluating the osseointegration of dental implants on a rabbit model treated with high-dose intravenous bisphosphonates in the long term and short term.

## 2. Materials and Methods

### 2.1. Study Design and Treatment

22- to 26-week-old female New Zealand White rabbits (3.2 kg to 4.2 kg) were randomly allocated into control and experiment groups, and each group was further divided into long-term and short-term subgroups with 5 rabbits in each subgroup (Table 1). Each rabbit was given zoledronic acid (experiment group, 0.1 mg/kg, s/c) or vehicle saline (control group, 0.1 mg/kg, s/c) three times per week for four weeks prior to surgery (animals underwent dental implant placement and tooth extraction. The tooth extraction was done for other investigation and will be presented in another article). The injection continued after the surgery until sacrifice. Animals in the short-term subgroups were sacrificed 4 weeks after surgery, and those in the long-term subgroups were sacrificed 8 weeks after surgery (Figure 1). In total, animals received 8 weeks and 12 weeks of saline or zoledronic acid in the short-term subgroups and long-term subgroups, respectively.

### 2.2. Dental Implant Insertion

All the implant placement was conducted under general anaesthesia. Heart rate, respiration rate, SpO_2_, and body temperature were recorded throughout the entire procedure.

The rabbit was placed in a prone position and shaved on the top of the head. The surgical site was disinfected, and a straight incision on the sagittal crest was performed. The calvaria was exposed after the subperiosteal dissection. Under continuous irrigation with sterile physiological 0.9% saline solution, a 3.5 mm craniotomy was performed with a rotating trephine burr and a round bur leaving dura mater intact, which was detached step by step from the inner table using first a small applicator and then a Freer periosteal elevator. A cylinder titanium implant (Straumann® SLA, 6 mm, Basel, Switzerland) with a diameter of 4.1 mm was inserted, leaving 2 mm of the implant intracranially. The extracranial part of the implant was covered with a resorbable membrane (Geistlich Bio-Gide®, 25 mm × 25 mm, Wolhusen, Switzerland). The scalp was closed after the epicranial aponeurosis was repositioned and closed over the membrane with single interrupted sutures (Ethilon®). The sutures were removed after 2 weeks. Postoperative care including pain control and food care were given under guidance.  Figure 2 briefly introduced the steps of the procedure.

### 2.3. Fluorochrome Labeling

Three different fluorochrome labeling solutions were prepared and injected in sequence subcutaneously [12, 13]: calcein green (10 mg/kg, Sigma-C0875), alizarin complexone (30 mg/kg, Sigma-A3882), and oxytetracycline (20 mg/kg, Sigma-O5875) at week 1, week 2, and week 3 after dental implant placement, respectively, in the short-term subgroups. For long-term subgroups which were sacrificed at week 8, these fluorochrome labeling solutions were injected at week 2, week 4, and week 6, respectively.

### 2.4. Sacrifice and Sample Collection

All animals were euthanized by intravenous injection of ketamine through the ear vein. Calvaria containing the dental implant was resected (with a margin of which was no less than 10 mm away from the implant) and was preserved in 10% neutral buffered formalin solution for further examinations.

### 2.5. Microcomputed Tomography (Micro-CT) Examinations

To evaluate the bone volume, bone mineral density (BMD), and microarchitecture, all the samples were subjected to a microcomputed tomography (micro-CT) scanning (Skyscan1076; Bruker, Kontich, Belgium) at 88 kV and 100 *μ*A intensity with a resolution of 17.3 *μ*m pixel. The reconstruction data were quantitatively analyzed with the CT analyzer software (version 1.9; Skyscan, Kontich, Belgium).

The region of interest (ROI) was selected as the circular bone tissue around the implant from the surface of the dental implant to the distance of 1.5 mm away from the implant centered on the midline of the trabecular area on the horizontal level (Figure 3). Data of BMD, BV (bone volume), TV (tissue volume), BV/TV (bone volume fraction, BV/TV = bone volume/tissue volume [13, 14]), Tb.Th (trabecular thickness, 3D measures of the average thickness of the cancellous bone structure [14–15]), Tb.N (trabecular number, the number of trabecular plates per unit length [14–16][14–16][14–16][14–16][13–15]), and Tb.Sp (trabecular separation, average diameter of the marrow cavities from ROI) were extracted for statistical analysis.

After micro-CT analysis, the undecalcified specimens were embedded in Technovit® 9100 PMMA and later prepared to ground sections for fluorochrome labeling analysis and histological examinations with a final thickness of approximately 40-50 *μ*m. Each section was made in the same manner, and each specimen was able to make 2 optimal sections.

### 2.6. Fluorochrome Labeling Analysis

Fluorochrome labeling analysis was performed to analyze bone growth rate and the dynamic bone formation using the Zeiss LSM 710 Upright Confocal Microscope and the Zeiss LSM 780 Inverted Confocal Microscope (Zeiss, Oberkochen, Germany). Images analysis was performed using the ZEN 2012 software. Bone growth rates were calculated by dividing the measured average distance between two sequenced fluorochrome labeling lines by the interval days between two injections [13].

### 2.7. Histological Examinations

After laser confocal imaging, the sections were stained with 1% toluidine blue in 60*°*C water bath for 40 minutes and mounted with Permount® after complete air-dry overnight (37*°*C). Microscope images were taken using the Nikon Eclipse LV100 POL (Nikon, Tokyo, Japan).

Osseointegration assessment was conducted by measuring the bone-to-implant contact (BIC), which was calculated as the percentages of mineralized bone in direct contact with the implant surface. Images were analyzed using ImageJ image analysis system (ImageJ 1.33u; National Institutes of Health, Bethesda, MD) to measure the BIC quantitatively according to the protocol described in the previous studies [17–19]. BIC on both sides of the dental implant in both cortical and cancellous calvarial bone [20] was measured and subjected to statistical analysis.

### 2.8. Statistical Analysis

The IBM SPSS statistics software (version 24.0, IBM Crop, Armonk: NY, USA) was used to perform the statistical analysis. Comparison of BMD, microstructure, bone growth rates, and incidence of osteonecrosis between groups was performed by independent *t*-test at a significance level of 0.05. The analysis was reviewed by an independent statistician.

## 3. Results

### 3.1. Clinical Observations

All animals recovered well and went through the whole experiment uneventfully except for one in the ZA long-term group was found dead on the next day following surgery. All surgical sites healed well. No signs of infection, inflammation, or dehiscence were observed. Sutures were removed uneventfully two weeks postoperation.

### 3.2. Micro-CT Assessment

The 3D micro-CT images were reconstructed from region of interest (ROI) (Figure 4). The results of BMD and other bone microstructure indices representing implant osseointegration were analyzed using independent sample *t*-test (version 24.0, IBM Crop, Armonk: NY, USA). The results were summarized in Table 2. The intergroup comparison showed that in the ZA long-term subgroup, BV/TV, BMD, Tb.N, and Tb.Sp values were higher than that in the control long-term subgroup; however, the differences were not statistically significant (Figure 5). Similarly, no significant differences were found in comparison between the ZA short-term group and the control short-term group.

### 3.3. Fluorochrome Labeling Analysis

The distances between two sequenced fluorochrome labeling were measured. The average bone growth rates were calculated by dividing the amount of days in between the two sequenced fluorochrome labeling solution injections (Figure 6). In general, ZA-treated group (both at week 4 and week 8) demonstrated significant reduced bone growth rates compared to control counterparts in all time intervals (weeks 1-2, weeks 2-3, weeks 2-4, and weeks 4-6) (Table 3, Figure 6). In the intragroup comparison, the averaged bone growth rates in each subgroup were used. Significant lower bone growth rates in the ZA short-term subgroup (from week 1 to week 3) were seen compared to ZA long-term subgroup (from week 2 to week 6), while no significant difference was detected between control long-term and control short-term subgroups (Figure 7).

### 3.4. Histomorphological Analysis

Histological images demonstrated comparable mineralization along the dental implant surface on both sides in both groups (Figure 8). The results of BIC were measured using the 10x objective of the microscope and are summarized in Table 4. Statistical analysis is shown in Figure 9. Significant lower BIC was found in ZA-treated animals compared to controlled animals at week 4, but then it increased to a level that was slightly lower than their control counterparts at week 8, and the difference at the later time point was found not significant at statistic level. When results were compared to intragroup, no significant difference was detected in neither the control group nor the ZA group.

## 4. Discussion

The understanding of the effect of high-dose BPs on osteointegration of dental implant is very limited. Clinicians desire to have more evidence on whether the success rates of dental implant therapy are affected in patient receiving high-dose BP treatment.

BPs were found to decrease bone turnover rates and thus increase bone mineral density significantly in osteoporotic patients in the first year of treatment and then reaches a plateau [21–22]. Similar findings were reported in animal studies which showed increased BMD, BV/TV, and Tb.Th, in osteoporotic animals (induced by ovariectomy surgery) treated with BPs [23–25]. Our previous studies showed significantly increased bone mineral density in ovariectomized animals treated with BPs [26–28]. In another animal study [29] using a tumor model, significant increase in BMD, BV/TV, Tb.Th, and Tb.N were detected in tumor-bearing animals treated with BPs, whereas in the control healthy animals, BP treatment did not significantly change the bone mineral density and other trabecular architecture.

In the present study, animals in the long-term ZA group demonstrated increase in BV/TV, Tb.Th, and BMD, but not statistically significant when compared with that in the control group. In the short-term ZA group, BV/TV, BMD, and Tb.N showed slight increase as well; however, Tb.Th declined slightly in comparison with that in the control group. This result may be due to the nonsignificant effect of BPs on normal bone tissue in accordance with the previous mentioned findings. Secondly, these parameters relate closely to the trabecular bones, which are comparatively much less in calvarial bones than in long bones, therefore makes the calculated results less variant. However, measures have been done to minimize the interference of cortical bones: ROI was selected centered on the midline of the trabecular zone horizontally. Another reason would be the relatively small sample size of this study. Lastly, the artifact caused by the metal implant may also affect the accuracy of the results.

Bone growth rates of the calvarial bone dropped significantly when animals were treated with BPs both long-termly and short-termly in the present study. The reduced bone growth rates mean reduced new bone formation, which is in conformity with the findings in other studies concerning the mechanism of bisphosphonate actions [30–33]. The decreased bone formation caused by BPs may be explained why BV/TV and BMD showed no significant increase even when high doses of BPs were given in our study. However, the reduced bone formation does not seem to relate to the diminished osteoblastic activity, which was suspected to be caused by the application of BPs. Actually, many studies described an improved proliferation of osteoblasts [1, 34, 35] and an inhibitory effect on apoptosis of osteocytes and osteoblasts [36, 37]. Therefore, this bone formation reduction was thought to respond to the declined bone resorption and the following diminished bone remodeling.

Initially at week 4, BIC was found significantly lower in the ZA-treated animals compared to controlled animals; it may reveal an adverse effect of ZA on osseointegration in the short term. However, BIC demonstrated a gain from week 4 to week 8 (though not statistically significant), to a level that was similar though slightly lower than the control counterparts; in the meantime, BIC decreased in the control group from week 4 to week 8. The gain of BIC in ZA group may be related to the significantly higher bone growth rates in the ZA long-term group compared to ZA short-term group. At week 8, BIC in the ZA group showed no significant difference in comparison with the control group. This result suggests that ZA may have an unfavorable effect on osseointegration in the short term. However, this effect seemed to diminish in the long term. How the BIC will change in the longer-term needs further investigations.

Currently, a history of oral or intravenous BP use is not considered an absolute contraindication for dental implant insertion. Osseointegration of dental implants was not significantly affected in these patients according to a systematic review [38]. However, current available studies are of levels III to II, which are not strong enough to support any conclusions.

Ayan et al. [39] reported a significant increase of BIC in tibia at week 2 and week 4 after a single dose of systemic ZA in rabbit model. In another animal study [40], implants were placed in the tibia of ovariectomized rabbit, and systemic ZA (single-dose infusion) was demonstrated to improve osseointegration as well. Similar results were reported in other studies [40–42]. These animal studies varied in BP type, dosage, and route of administration, and the implants were placed in the tibia, which exhibited a lower remodeling rate than that in jaw bones.

Different results were observed in animal studies that placed implants in jaw bones. Using an ovariectomized rat model with implant placement in mandibles, Cardemil et al. [43] demonstrated a significantly lower BIC in the ZA group (single IV dose) compared to control group at 14 days. The BIC showed some growth to a level higher than the control counterparts at 28 days and exhibited no significant difference at this time point. The results in our study were similar except that the reduction in BIC was not significant in the ZA group at the early time point though the dosage of ZA was much higher in our study. In another study placing implants in the parietal bone of rabbit [44], it was concluded that systemic use of alendronate may delay the osseointegration of the newly formed bone.

The results of the BIC may be interpreted in a way that BPs may have an adverse effect on osseointegration in calvarial bone in the short term but this effect tends to diminish or possibly become a positive effect in the long term. However, this interpretation has to be considered with care due to the limited number of animals included in each group. In addition, rabbits exhibit a different composition of bone and a much higher bone turnover rate than human, and translation of the results of rabbits to human subjects needs critical assessment.

In conclusion, high-dose ZA treatment inhibits bone growth rates and showed an adverse effect on osseointegration of dental implant in short term. However, no significant effect on bone mineral density or trabecular microarchitecture is detected in the rabbit model with implant placement on the calvarial bone.

## Figures and Tables

**Figure 1:** Timeline of the study. The baseline is set at the implant insertion day after 4 weeks of vehicle or ZA treatment. Sacrifice time points include 4 weeks and 8 weeks after implant insertion.

**Figure 2:** Surgical procedures of dental implant placement. (a) Straight incision on the sagittal crest is performed; (b) the epicranial aponeurosis is carefully dissected from the scalp to use it later for covering the dental implant; (c) after the subperiosteal dissection, the calvaria is exposed; (d) a 3.5 mm craniotomy is created with a trephine burr and a round burr leaving the inner table intact. Through this hole, the underlying dura is detached from the inner table using a small applicator and a Freer periosteal elevator; (e) a cylinder titanium implant (Straumann® SLA, 6 mm, Basel, Switzerland) is inserted, leaving 2 mm of the implant extracranially (f); (g) the extracranial part of the implant was covered with a resorbable membrane (Geistlich Bio-Gide®, 25 mm × 25 mm, Wolhusen, Switzerland); (h) the epicranial aponeurosis was closed over the membrane with single interrupted sutures (Ethilon®); (i) the wound was closed with single interrupted sutures.

**Figure 3:** The region of interest (ROI) is selected from the surface of the dental implant to the distance of 1.5 mm away from the implant ((a) red area, cross section view) centered on the midline of the trabecular area on the horizontal level ((b) red line, frontal view). In total, 61 layers are selected.

**Figure 4:** The 3D model of each specimen is generated from the region of interest (ROI) defined in this study.

**Figure 5:** Intergroup comparison of BMD, BV/TV, Tb.Th, Tb.N, and Tb.Sp in the calvarial bone between control and ZA-treated groups at the time point of week 4 and week 8. No significant difference is detected in all the assessed parameters.

**Figure 6:** (a) Fluorochrome labeling analysis at week 4 is performed using 10x objective of Zeiss LSM 710 Upright Confocal Microscope, and upper images are stitched after using the tile scan function of the Zeiss LSM 780 Inverted Confocal Microscope. (b) Fluorochrome labeling analysis at week 8 is performed using 10x objective of Zeiss LSM 710 Upright Confocal Microscope, and upper images are stitched after using the tile scan function of the Zeiss LSM 780 Inverted Confocal Microscope.

**Figure 7:** Intergroup comparison and intragroup comparison of bone growth rates (*μ*m/day) of the calvarial bone. CS: control short-term subgroup; ZS: ZA short-term subgroup; CL: control long-term subgroup; ZL: ZA long-term subgroup. ^∗∗∗^*P* < 0.001.

**Figure 8:** Histological assessment for the control and ZA-treated groups at week 4 is illustrated in the picture (2x objective), and measurement of bone-to-implant contact (BIC) is made using the 10x objective on both sides of the implant. Histological assessment for the control and ZA-treated groups at week 8 is illustrated as above (2x objective), and measurement of bone-to-implant contact (BIC) is made using the 10x objective on both sides of the implant. Comparable mineralization is shown in both groups and at different time points.

**Figure 9:** Intergroup and intragroup comparison of BIC in the calvarial bone. Significant difference is detected in the comparison between control group and ZA group at week 4 but not at week 8. In the intragroup comparison, no significant difference is found. ^∗^*P* < 0.05.

**Table 1:** Group allocation and treatment.

Groups	No.	Treatments	Sacrifice
Control	5	Veh+implant insertion	Week 4
	5	Veh+implant insertion	Week 8
Experiment	5	ZA+implant insertion	Week 4
	5	ZA+implant insertion	Week 8

Veh: vehicle saline; ZA: zoledronate acid.

**Table 2:** Statistical analysis result of bone mineral density (BMD) at the calvarial site and other bone microstructure indices (mean ± SD).

Groups	Control short-term	Control long-term	ZA short-term	ZA long-term	*P* value^∗^	*P* value^∗∗^
Parameters						
BMD	0.63 ± 0.08	0.61 ± 0.07	0.66 ± 0.05	0.63 ± 0.02	0.593	0.546
BV/TV	0.56 ± 0.07	0.50 ± 0.07	0.55 ± 0.06	0.52 ± 0.03	0.776	0.638
Tb.Th (mm)	0.112 ± 0.012	0.106 ± 0.009	0.105 ± 0.002	0.106 ± 0.004	0.215	0.992
Tb.N (1/mm)	5.00 ± 0.42	4.71 ± 0.30	5.25 ± 0.64	4.93 ± 0.42	0.490	0.394
Tb.Sp (mm)	0.11 ± 0.02	0.12 ± 0.02	0.12 ± 0.03	0.13 ± 0.02	0.425	0.358

^∗^ *P* value between control group and ZA group at week 4. ^∗∗^*P* value between control group and ZA group at week 8. BMD: bone mineral density; BV/TV: bone volume/tissue volume, bone volume fraction; Tb.Th: trabecular thickness; Tb.N: trabecular number; Tb.Sp: trabecular separation.

**Table 3:** Bone growth rates measured by fluorochrome labeling analysis (mean ± SD).

Group statistics	Bone growth rates (*μ*m/day)			*t*-test
	Groups	*N*	*Mean* ± *SD*	Sig. (2-tailed)^∗^
Weeks 1-2	CS	5	2.68 ± 0.25	0.000
	ZS	5	1.10 ± 0.03	
Weeks 2-3	CS	5	1.85 ± 0.17	0.000
	ZS	5	0.86 ± 0.08	
Weeks 2-4	CL	5	2.45 ± 0.22	0.000
	ZL	4	1.77 ± 0.11	
Weeks 4-6	CL	5	1.85 ± 0.23	0.000
	ZL	4	0.99 ± 0.13	

CS: control short-term group; ZS: ZA short-term group; CL: control long-term group; ZL: ZA long-term group. ^∗^*P* value.

**Table 4:** Bone-to-implant contact (BIC) in calvarial bone at week 4 and week 8.

Group	Week 4			Week 8			*P* value^∗^
	*N*	Mean	SD	*N*	Mean	SD	
Control	5	0.38	0.035	5	0.35	0.063	0.401
ZA-treated	5	0.28	0.083	4	0.34	0.019	0.151
*P* value^∗∗^	0.030			0.815			

^∗^Intragroup comparison between two time points. ^∗∗^Intergroup comparison between control and ZA-treated groups.

## Data Availability

The data used to support the findings of this study are included within the article.

## Abbreviations

ZA: Zoledronic acid
Micro-CT: Microcomputed tomography
MRONJ: Medication-related osteonecrosis of the jaws
BP: Bisphosphonate
BMD: Bone mineral density
BV: Bone volume
TV: Tissue volume
BV/TV: Bone volume fraction
BV/TV: Bone volume/tissue volume [14]
Tb.Th: Trabecular thickness
Tb.N: Trabecular number
Tb.Sp: Trabecular separation
ROI: Region of interest
BIC: Bone-to-implant contact.
